# Diagnosis of Alzheimer's Disease by Time-Dependent Power Spectrum Descriptors and Convolutional Neural Network Using EEG Signal

**DOI:** 10.1155/2021/5511922

**Published:** 2021-04-24

**Authors:** Morteza Amini, Mir Mohsen Pedram, AliReza Moradi, Mahshad Ouchani

**Affiliations:** ^1^Department of Cognitive Modeling, Institute for Cognitive Science Studies, Shahid Beheshti University, Tehran, Iran; ^2^Department of Electrical and Computer Engineering, Faculty of Engineering, Kharazmi University, Tehran, Iran; ^3^Department of Cognitive Modeling, Institute for Cognitive Science Studies, Tehran, Iran; ^4^Department of Clinical Psychology, Faculty of Psychology and Educational Science, Kharazmi University, Tehran, Iran; ^5^Department of Cognitive Psychology, Institute for Cognitive Science Studies, Tehran, Iran; ^6^Institute for Cognitive and Brain Science, Shahid Beheshti University, Tehran, Iran

## Abstract

Using strategies that obtain biomarkers where early symptoms coincide, the early detection of Alzheimer's disease and its complications is essential. Electroencephalogram is a technology that allows thousands of neurons with equal spatial orientation of the duration of cerebral cortex electrical activity to be registered by postsynaptic potential. Therefore, in this paper, the time-dependent power spectrum descriptors are used to diagnose the electroencephalogram signal function from three groups: mild cognitive impairment, Alzheimer's disease, and healthy control test samples. The final feature used in three modes of traditional classification methods is recorded: *k*-nearest neighbors, support vector machine, linear discriminant analysis approaches, and documented results. Finally, for Alzheimer's disease patient classification, the convolutional neural network architecture is presented. The results are indicated using output assessment. For the convolutional neural network approach, the accurate meaning of accuracy is 82.3%. 85% of mild cognitive impairment cases are accurately detected in-depth, but 89.1% of the Alzheimer's disease and 75% of the healthy population are correctly diagnosed. The presented convolutional neural network outperforms other approaches because performance and the *k*-nearest neighbors' approach is the next target. The linear discriminant analysis and support vector machine were at the low area under the curve values.

## 1. Introduction

The term “dementia” refers to many neurodegenerative illnesses caused by neuronal failure and death that interrupt cognitive and behavioral activities. The most prevalent of the several types of dementia is Alzheimer's disease (AD), with about 70% of worldwide dementia cases. It affects the individual over 65 years, and the rate of occurrence increases exponentially at the age of 65 years [1–3]. To date, AD has not been resolved by palliative therapies, which have been temporarily slow to deteriorate in patients and caregiver living [4]. Today, only postmortem diagnosis of definitive AD is possible after examining the structural brain injury that is typical of the condition. Accuracies of up to 90% have usually been recorded for modern testing procedures, such as neurological assessments and medical history. The National Institute on Aging and Alzheimer's Association has established the existing standards of clinical diagnosis of AD, and the Alzheimer's Association has established them [5]. These standards are an advancement in the previous guidelines, which had been developed in 1984 by the National Institute of Neurological And Communicative Diseases and Stroke/Alzheimer's Disease and Related Disorders Association (NINCDS-ADRDA) [6]. It is part of the NINCDS-ADRDA guideline. These revised suggestions require neuroimagery and the use of biomarkers and cerebrospinal fluid to diagnose AD for symptomatic people [5].

A guideline for diagnosing and monitoring AD [7] was established by the European Federation of Neurological Societies. The Mini-Mental State Assessment [8, 9] is the most used AD diagnosis method to test cognitive ability. The revised Montreal Cognitive Assessment [10] is commonly used in therapeutic functional applications and the revised Addenbrooke Cognitive Evaluation [11]. Another example of neurological testing is the Extreme Cognitive Disorder, Alzheimer's Cognitive Disease Evaluation Scale, Neuropsychological Assessment Battery, and Serious Impairment Battery. The Trail Making Test [12] and the clock drawing test [13], by contrast, focus not only on testing thinking abilities but also on concentrating and administrative work. In comparison, the visual learning test and the Rey Auditory Fluency Assessment assess all patient support practice skills [14]. In some instances, AD is also associated with other diseases that cause dementia as brain vascular injury, Lewy body disease, and Parkinson's disease [15]. The early diagnosis of AD and these problems is improved using methods that gain biomarkers as early signs overlap [16–19]. Electroencephalogram (EEG) is a technology that enables the recording by postsynaptic potentials of a thousand neurons of identical spatial orientation of the time of cerebral cortex electrical activity. Scalp-positioned electrodes measure the electrical potentials. EEG's spatial resolution refers to the number and location of electrodes on the scalp. The most used configuration is the international 10-20 system, which consists of 21 electrodes; the 10-20 system is often used for higher density versions, for instance, 10-10 and 10-5, usually 64 and 128 electrodes, and the Maudsley [20] and geodesic positions [21] alternating layouts. Reliable therapeutic methods have been shown in recent years for the diagnosis and analysis of disorders and cortical conditions like the Huntington syndrome, the autism spectrum disorder [22], epilepsy and seizure [23], brain ischemia [24], frontotemporal dementia [25], and Parkinson's dementia [26]. Furthermore, EEG evaluations were carried out on the comparative diagnosis of AD and other dementia-contributing diseases such as brain vascular injuries [27, 28] and Lewy disease [29, 30]. Theta (*θ*) 4–8 Hz, delta (*δ*) 0.1–4 Hz, beta (*β*) 12–30 Hz, alpha (*α*) 8–12 Hz, and gamma (*γ*) > 30 Hz are typically divided between 5 major frequency bands in the analytics. Also, more divisions into these bands (high alpha, low alpha, low beta) are considered, but the subband frequency limits are not uniform in all studies. The different data on brain function and synchronization are given in each frequency band [31–33]. There has been a comprehensive study of the possible use of electroencephalography to diagnose dementia and AD [34]. EEG is a high time resolution noninvasive, comparatively inexpensive, and potentially mobile technology (about milliseconds). It was studied primarily as an AD diagnostic tool when comparing EEG records in AD patients with control subjects (healthy individuals) [35, 36]. AD is generally known to decrease the complexity of EEG signals and synchronous change in EEG.

These improvements have been used as discriminatory features for AD diagnosis in EEG recordings. Several methods of assessing the complexity of EEG signals have been established. The connection factor and the first positive exponent of Lyapunov have been used frequently [37–42]. EEG signals from AD patients have been shown to show lower (lower complexity) values of certain tests than signals from age-matched control subjects. Other information-theoretical methods, in specific entropy-based approaches, have appeared as theoretically useful EEG indicators for AD: epoch-based entropy [43, 44], sample entropy [45], Tsallis entropy [46], approximate entropy [47, 48], multiscale entropy [49], and complexity of Lempel-Ziv [50]. These approaches relate the strength of a signal to unpredictability: irregular signals are more complicated than regular ones because they are erratic. Different detection algorithms have been suggested in previous studies for epileptiform EEG data [51]. Current seizure detection methods use hand-built feature extraction techniques from EEG signals [52], including frequency domain, time domain, time-frequency domain, and nonlinear evaluation of signals [53, 54]. The features selected must be listed after the feature extraction to identify various EEG signals using all forms of classifiers [55]. Hamad et al. employed a differential wavelet transformation procedure to obtain the feature collection, then trained the radial reference algorithm with the support vector machine (SVM), demonstrating an epilepsy diagnosis with the suggested SVM gray wolf optimizer [56]. For the refinement of the SVM parameters based on genetic algorithms and particle swarm optimization, Subasi et al. developed a hybrid model. The proposed SVM hybrid model shows that neuroscientists use EEG as an essential method for diagnosing epileptic seizures [57]. However, the manual function selection criteria are not eradicated by these strategies [58]. The feature extraction is an important stage in classification determination, as it determines its specificity in large part. A system for classifying without the removal of complicated properties was suggested. Furthermore, recent advancements in deep learning have shown a new way of coping with this problem. Deep learning has in recent years reached the recognized form of computer vision and machine learning and has demonstrated that almost all human and superhuman functions such as pattern recognition and sequence learning perform numerous functions [59], among other things. Feature extraction before classification is more advantageous than entering raw EEG samples directly into the classifier. Nevertheless, several recent research types have not performed feature extraction, but instead, raw EEG signals were used for the deep learning model [60, 61].

In this paper, the time-dependent power spectrum descriptor (TD-PSD) method is utilized for feature extraction of the EEG signal from three categories of MCI, AD, and HC sample test. The final feature with labeling is used in three types of traditional classification methods, including *k*-nearest neighboring (KNN), SVM, and linear discriminant analysis (LDA) approaches, and the results are recorded. Finally, an architecture of convolutional neural network (CNN) for AD patients' classification is provided. The results are indicated using performance analysis.

## 2. Literature Review

EEG signals' complex and nonlinear nature implies creating new methods to study machine and signal processing [62, 63]. Recent progress has been made to enhance high-level abstractive methods for the automated removal of complex data features in the field of deep learning methodologies [64–66]. In the last years, these deep learning methods are usually used in image processing, natural language processing [67–70], speech processing, and video games [71]. The biomedical area has also been identified with these methods [72–74]. Acharya et al. [60] suggested a deep, 13-layer neural CNN that distinguishes normal, preictal, and EEG signals of seizure. In the study, 300 EEG signals were used for registering a classification rate of 88.67%. The same group proposed a deep neural network approach for an innovative EEG-based depression screening method [60]. This investigation's outcomes are reported in 15 regular and 15 depressive patients, 93.5% (left hemisphere) and 96.0% (right hemisphere). Oh et al. [75] suggested that further studies used EEG signals to diagnose Parkinson's disease. A 13-layer CNN model of 20 healthy and 20 Parkinson patients reached an accuracy of 88.25%. Hong et al. [76] propose a mathematical model employing Long Short-Term Memory (LSTM), a recurrent neural network (RNN) that predicts the mild cognitive impairment of AD. The data is taken in image form in this research, and the preprocessing is done by skull strip, normalization, registration, smoothing, and segmentation. The training is carried out by feeding sequential data with time steps to the model after preprocessing, and the model projects the state of the next six months. During model testing, when the feature data for the 18th and 24th months is presented, it forecasts the state of the subject for the 30th month. Similarly, Aghili et al. [77] suggest an RNN approach to evaluate longitudinal data to differentiate between stable people against AD individuals. The input is preprocessed, and the function is normalized. It is fed into LSTM and gated recurring units after preprocessing the data. In the model of LSTM and gated regular units, each subject's time point data is provided to the corresponding cell along with its final diagnosis mark to learn the pattern of data transition. The effect models are contrasted with the effects of nonrecurrent networks, i.e., multilayer perceptron (MLP), for all data arrangements. For each patient, the data is fed into the MLP once. There are many trainable parameters in the LSTM models that need to be substantially trained for sequential data and are vulnerable to overfitting the training data. The purpose of unsupervised feature learning is to define AD using the principle of unsupervised feature learning. An approach used sparse filtering to learn the expressive characteristics of brain images [78]. The SoftMax regression is trained to classify the circumstances. In the first step, there are three phases: sparse filtering is trained, and its W weight matrix is calculated. The sparse filtering learned is used to extract from each sample the local characteristics. In terms of negative matrix factorization (NMF) and SVM with limitations of certainty, Padilla et al. [79] offer a novel conclusion technique for the early determination of Alzheimer's disease. Through implementing the Fisher discriminant proportion and non-NMF for highlighting preference and extraction of the most important highlights, the single-photon emission computed tomography and positron emission tomography datasets are studied (see Table 1).

## 3. Research Methodology

The proposed study uses the EEG signal to describe the phases of the disorder. It is suggested that a deep CNN network architecture is learned to distinguish multichannel human EEG signal data into different stages and that increases the efficiency of classification. This work includes the modules below:

- Preprocessing
- Feature extraction
- Classification

### 3.1. Feature Extraction

The EEG trace is expected to be explicated in a function of frequency *X*[*k*], using the discrete Fourier transform, as a product of the sampled representation of the EEG signal as *x*[*j*] with *j* = 1, 2, ⋯, *N*, length *N*, and sampling frequency fs (Hz). Parseval's theorem explains that the function's total square is the complete square of its transformation; the process starts with the extraction of features.

(1) $$\begin{array}{c} \overset{N-1}{\underset{j=0}{\sum }}{\left|x\left[j\right]\right|}^{2}=\frac{1}{N}\overset{N-1}{\underset{k=0}{\sum }}\left|X\left[k\right]X^{*}\left[k\right]\right|=\overset{N-1}{\underset{k=0}{\sum }}P\left[k\right]. \end{array}$$

According to the above equation, *P*[*k*] is the phase-excluded power spectrum. It means that the frequency index is obtained by multiplying*X*[*k*]by the*X*^∗^[*k*]conjugate divided by*N*, where the phase-excluded power spectrograph is *P*[*k*], i.e.,*X*[*k*]has its conjugate *X*^∗^[*k*], separated by *N*, which is compounded by*k*, and frequency index. The full definition of the frequency as obtained by the Fourier transform is usually well-known to be symmetrical concerning zero frequency; i.e., it has similar sections extending to the frequencies, which are both positive and negative [89]. The whole spectrum, including positive and negative frequencies, is free from this symmetry. Access to spectral power from the time domain has not been completed. According to the concept of a one-minute *m* of the order *nP*[*k*] of the power spectral density, all irregular moments are also zero by the frequency distribution model's statistical approach.

(2) $$\begin{array}{c} m_{n}=\overset{N-1}{\underset{k=0}{\sum }}k^{n}P\left[k\right]. \end{array}$$

In the latter equation, the Parseval theorem of Equation (1) may be used where *n* = 0 is used, and the Fourier transform time-differentiation feature for nonzero quantities of *n* is used. Such a feature explicitly indicates the*n*^′th^equal to multiply the*k*augmented by the spectrum to the*n*^′th^power, the derivative of a time-domain function referred to as∆^*n*^for various time signals.

(3) $$\begin{array}{c} F\left[{∆}^{n}x\left[j\right]\right]=k^{n}X\left[k\right]. \end{array}$$

To this end, as seen in Figure 1, the description of the characteristics used is as follows:

*Root squared zero-order moment (* $\bar{m_{0}}$): this is a function that shows the overall power of the frequency domain and is as follows:

(4) $$\begin{array}{c} \bar{m_{0}}=\sqrt{\overset{N-1}{\underset{j=0}{\sum }}x{\left[j\right]}^{2}s}. \end{array}$$

All channels may also standardize their corresponding zero-order moments by dividing all channels into zero-order moments.

*Root squared second and fourth-order moments*: according to Hjorth [89], the second time is used as power, but then, a spectrum shifted *k*^2^*P*[*k*], referring to the frequency function:

(5) $$\begin{array}{c} \bar{m_{2}}=\sqrt{\overset{N-1}{\underset{k=0}{\sum }}k^{2}P\left[k\right]=}\sqrt{\frac{1}{N}\overset{N-1}{\underset{k=0}{\sum }}{\left(kX\left[k\right]\right)}^{2}}=\sqrt{\overset{N-1}{\underset{j=0}{\sum }}{\left(∆x\left[j\right]\right)}^{2}}. \end{array}$$

A repetition of this procedure gives the moment:

(6) $$\begin{array}{c} \bar{m_{4}}=\sqrt{\overset{N-1}{\underset{k=0}{\sum }}k^{4}P\left[k\right]=}\sqrt{\overset{N-1}{\underset{j=0}{\sum }}{\left({∆}^{2}x\left[j\right]\right)}^{2}}. \end{array}$$

The total energy of the signal is decreased by consideration of the second and fourth signals; thus, a power transformer is implemented to normalize the domain of *m*_0_, *m*_2_, and *m*_4_ to minimize the noise effect on all moment-based features as follows:

(7) $$\begin{array}{c} m_{0}=\frac{{\bar{{\text{m}}_{0}}}^{\lambda }}{\lambda },\\ m_{2}=\frac{{\bar{m_{2}}}^{\lambda }}{\lambda },\\ m_{4}=\frac{{\bar{m_{4}}}^{\lambda }}{\lambda }. \end{array}$$

The experimental setting of*λ*is 0.1. From these parameters, consequently, the first three features extracted are described as follows:

(8) $$\begin{array}{c} f_{1}=\log\left(m_{0}\right),\\ f_{2}=\log\left(m_{0}-m_{2}\right),\\ f_{3}=\log\left(m_{0}-m_{4}\right). \end{array}$$

*Sparseness*: this feature measures the amount of vector energy in just several more elements. It is followed as

(9) $$\begin{array}{c} f_{4}=\log\left(\frac{m_{0}}{\sqrt{m_{0}-m_{2}}\sqrt{m_{0}-m_{4}}}\right). \end{array}$$

A feature represents a vector with all elements equivalent to a zero-sparseness index, i.e., *m*_2_ and *m*_4_ = 0, due to differentiation and log(*m*_0_/*m*_0_) = 0, while it should require a value greater than zero for all other sparseness levels [90].

*Irregularity factor (IF)*: a measure that expresses the ratio of peak numbers divided by zero crossings. According to [91], only in terms of their spectral instances can the number of upward zero crossings (ZC) and the number of peaks (NP) in a random signal be specified. It is necessary to write the corresponding feature as

(10) $$\begin{array}{c} f_{5}=\frac{\text{ZC}}{\text{NP}}=\frac{\sqrt{m_{2}/m_{0}}}{\sqrt{m_{4}/m_{2}}}=\sqrt{\frac{m_{2}^{2}}{m_{0}m_{4}}}=\frac{m_{2}}{\sqrt{m_{0}m_{4}}}. \end{array}$$

*Covariance (COV)*: COV function is the ratio of the standard deviation on arithmetic averages as follows:

(11) $$\begin{array}{c} f_{6}=\log\left(\frac{\sqrt{\left(\sum_{j=0}^{N-1}{\left(x-\bar{x}\right)}^{2}\right)/n}}{\bar{x}}\right). \end{array}$$

*Teager energy operator (TEO)*: it mainly displays the magnitude of the signal amplitude and instantaneous changes that are very susceptible to minor changes. While TEO was proposed for nonlinear speech signal modeling, it was later used to process audio signals. It is formed as follows:

(12) $$\begin{array}{c} f_{7}=\log\left(\Psi \left(\text{x}\left[\text{j}\right]\right)\right)=\log\left(\overset{N-1}{\underset{j=0}{\sum }}x^{2}\left[j\right]-x\left[j-1\right]x\left[j+1\right]\right). \end{array}$$

In conjunction with the schematics in Figure 1, from each EEG record *x*, first, the seven features are extracted. In the classification method, the features described by the corresponding vector *f* are used. These characteristics can be assumed to reflect the EEG behavior in the form of cepstrum. Contrary to the well-known voice cepstral features [92], our EEG features have been obtained as the orientation between characteristics derived from a nonlinear EEG record and an initial EEG record following the equation. In the case of EEG classifications at differing levels of force, orientation-based feature extraction processes have recently been demonstrated to be of considerable significance for research on intact-limbed subjects as force generation relies on multiple hand muscle coordination [93].

There have not been any prior attempts to test the efficacy of specific features in amputees. In the coming subsection, the suggested orientation-based feature is adequate for amputees to classify EEG signals with different classes. In the remainder of the essay, the last feature *f* is defined, together with the time-dependent descriptor spectrum, from all channels, given as TD-PSD.

### 3.2. Convolutional Neural Network

CNN is one of the learning networks inspired by the MLP in this type of neural network. This deep network comprises an input layer, an output layer, and a deeply hidden layer. Firstly, the problem's signal or data are identified and trained into the algorithm. The hidden weights of the output layer appear in many forms [94]. If the algorithm output includes numerous numerical components, such as a binary number or index (e.g., signal classification, normal = 1, abnormal = 2), then the algorithm presented is a classification or detection algorithm. That is, the outcomes are weighted after the training of several signals. When a new signal is added to the algorithm other than the training signals, the signal form is identified, for example, whether a matrix of various kinds of signals is sent to the algorithm and trains the machine, signals of benign or malignant types of cancer, Alzheimer's, sarcoma, or brain tumor, for example. The type of disease can be identified by the algorithm with the weights obtained. CNN consists of numerous hidden sublayer forms that are explained as follows.

### 3.3. Convolutional Sublayer

The basic of the CNN is the convolutional sublayer, and it is possible to view its output matrix as a three-dimensional neuron matrix. For a deeper explanation of this, imagine traditional neural networks. Each layer was a little more than a list (one-dimensional as a rectangle) of neurons in regular neural networks in which each neuron generated its output, and gradually, a collection of outputs referring to each neuron was produced. However, instead of a single list, it is presented with a three-dimensional list (one cube) where the neurons are organized in three dimensions. Therefore, a three-dimensional matrix would also be the production of this cube. This principle and the distinction between the two are illustrated in the images below [95].

Let the size of the input matrix be 20 × 16 × 16. Thus, utilizing a receptive field of 3 × 3, each neuron would have 3 × 3 × 20 = 180 connections to the input matrix in the conventional layer. Notice that space's connection is local (for example, 3 × 3 here) but covers the maximum depth (Figure 2). An input displays the left image (for example, a 3 × 32 × 32 image). The neuron matrix is observed in the conventional blue sheet. In terms of spatial coordinates (length and width) in the input matrix, each neuron in the conventional layer is related to one local region only, but this connection extends in-depth (i.e., covers all color channels). There are depths (in this case, neurons) that all look at one place at the entrance.

The hyperparameter regulates the output matrix's dimension. The depth, stride, and zero-padding layer are these three parameters. The parameter can be used in the depth of the output matrix. This parameter regulates the number of neurons that bind to a region in the conventional layer's input matrix. This variable is analogous to multiple neurons in a hidden layer all attached to one input in classical neural networks. All these neurons learn to function on various feedback features in which the deep columns around the spatial dimensions must be defined (width and height). When the stride is equal to 0, the spacing coordinates of just five spaced points are allocated to a new depth column of neurons. Also, in large output matrixes, this leads to receptive areas of overlap between columns. Alternatively, the receptive areas are less frequent if the measures taken are bigger, and the output mass is smaller in the spatial dimension [96]. Overriding the inbound matrix with a zero pad is also more precise. In other terms, fill zero with the input picture circle. Our signal is put within a zero signal like inserting row 1 and column 2 at the beginning and end of a signal.

### 3.4. Max Pool Sublayer

One standard technique in conventional architecture is the positioning of a pooling layer between many successive layers. This layer's purpose is to minimize the matrix (input) size (width and height) by reducing the number of variables and calculations within the grid and thereby overfitting the monitor. The pooling layer functions and uses it on each depth cut of the input matrix independently. The MAX function resizes the spot. The most typical way to utilize this layer is to use this layer with filters of 2 × 2 sizes with phase *S* = 2 that eliminates any depth cuts at the input by deleting two elements from the width and two elements from the height and deleting 2% of the values [97].

### 3.5. Activation Function

Artificial neural networks' activation function determines the node's output node or “neuron” according to the input or group of inputs. In the next node, this output is known as the input. It follows before a solution to the issue is sought. The outcome values are translated to the target set, such as 0 to 1 or -1 to 1 (depending on the activation function selected). Using the logistic activation function, for example, transforms all inputs into true real ranges between 0 and 1. Another essential characteristic of an activation function is that it must be derivative to execute the optimization technique for backpropagation error and measure the weight gradient error in the network and use gradient descent or another optimal approach. Another optimization is optimizing weight to reduce weight. The rectified linear unit (ReLU) is used in this paper for the use of functions as follows:

(13) $$\begin{array}{c} f\left(x\right)=\left\{\begin{array}{c} 0,\;x<0,\\ x,\;x\geq 0. \end{array}\right. \end{array}$$

Some activation functions are also not unique to a single variable and refer to the vector or different variables used in this article, such as SoftMax [98]:

(14) $$\begin{array}{c} f_{i}\left(\vec{x}\right)=\frac{e^{x_{i}}}{\sum_{j=1}^{J}e^{x_{j}}}. \end{array}$$

Also, to normalize input results, a batch normalization layer is applied to the network to speed up the training process and reduce network sensitivity between convolutional layers and nonlinearities. Also, to create an abnormal signal augmentation, a dropout layer on the fully connected layers is applied. Fully connected layers are used at the end of the hidden layer, which has been known to distinguish signals. The deep learning layer's outcome leads to a fully connected layer that drives the final classification judgment.

### 3.6. Receiver Operating Characteristic (ROC) Curve

In 2004, the ROC curves were developed, which were used to detect a radio noise signal [99]. These curves have recently been discovered to have important uses in medical decision-making. Presume having two kinds of individuals, one is normal and the other is a patient. It is a screening test on both our patients and healthy people, and the spectrum of values from the test ranges from 0 to the large number scale. In this case, the greater the test outcome, the greater the risk of the disease. (For certain things, the action can be the opposite.)

The ROC curve is established by the true-positive rate (TPR) projection in different threshold settings against the false-positive rate (FPR). The TPR is often identified in ML as sensitivity, recall or detection probability. Beginning from the ROC's left side, both the FPR and the TPR are zero at this point. (This argument indicates that the threshold line, which is the most significant number of test outcomes, is very large.) The TPR and FPR values in this case are measured and the next curve is drawn. The definition of TPR equals TP/Y, and the definition of FPR equals FP/N.

For a reduced number of previous values, let us reduce the threshold line. For lower values, the trend is replicated and eventually reaches the rightmost point of the ROC curve, which is equal to the baseline of the lowest value of the test outcome in this case. In this function, there is one TPR and one FPR. Accuracy relies entirely on allocating random errors and does not correspond with the real value or the value specified. In terms of bias, correctness is conveyed. A complete structural error can consist of one or more components of a systematic error. In the comparison value, a strong bias implies a large disparity. The two variables' sensitivity and specificity in statistics were used to determine the binary classification outcome (duality). When the data can be broken into positive and negative classes, using sensitivity and attribute indicators, the consistency of a test's outcomes that separate the information into these two divisions is observable and descriptive. Sensitivity means the number of positive cases that would be accurately checked as positive. Specificity means the number of negative cases that accurately label them as negative (positive = special illness, negative = other cases).

*True positive (TP)*: the positive signal is accurately detected.

*False positive (FP)*: the negative signal is detected with mistakes.

*True negative (TN)*: the negative signal is detected accurately.

*False negative (FN)*: the positive signal is detected with mistakes.

The sensitivity divides TP cases into the sum of true-positive and false-negative cases in statistical terms.

(15) $$\begin{array}{c} \text{Sensitivity}=\frac{\text{TP}}{\text{TP}+\text{FN}}. \end{array}$$

The confusion matrix is the role of the algorithms described in the field of artificial intelligence. Usually, for supervised learning algorithms, such a demonstration is being used, but it is often utilized in unsupervised learning. An instance of the predicted value is seen in each column of the matrix. Suppose it includes an actual (true) instance in each row. This matrix's name is also gained, making it possible to mistake and mess with the results. This matrix is commonly called a contingency matrix or an error matrix outside of artificial intelligence.

## 4. Results and Discussion

### 4.1. Data Collection

Multichannel EEG signals were captured using earlobe-electrode hallmark monopolar connections [100]. The location of the electrodes over the scalp was obtained according to the 10-20 International Electrode Positioning Method (i.e., Fp1, Fp2, F7, F3, Fz, F4, F8, T3, C3, Cz, C4, T4, T5, P3, Pz, P4, T6, O1, O2). In Figure 3, an example of EEG electrode placement is shown. The electrodes calculate the weak electrical potential in the microvolt range produced by brain activities. Recordings were conducted with closed eyes in a sleeping state. In this way, multiple brain regions can be believed to be governed by the exact hierarchical mechanism.

Data with a signal length of 300 seconds and a sampling frequency of 1024 and 256 samples per second were obtained. Just 180 seconds is extracted for each signal (i.e., from 60 to 240 seconds) to minimize the EEG context artifacts and convert each one to 256 samples per second. The sampling frequency, or sample rate, is the number of equal-spaced samples per unit of time. For instance, if there are 1024 equally spaced observations per second, the sampling rate is 1024/second or 1024 Hz. In this paper, for each second, 256 samples are used. Therefore, the length of the time series is 300∗256 = 76800. Moreover, the time interval from 60 to 240 seconds (of 300-second signals) is used with length 240 − 60 = 180. Finally, the length of the signal is 180∗256 = 46080. To summarize, the EEG capacity of human samples belonging to three categories has been recorded:

1. Patients who have Alzheimer's disease (AD)
2. Patients who suffer from mild cognitive impairment (MCI)
3. Healthy control (HC)

Figure 4 gives an example of extracted EEG recordings of 256 samples for each group.

Figures 5–7 show each category's time-frequency analysis based on continuous threshold wavelet transform. The EEG signal processing strategies are addressed in this section to extract the necessary quality information from clinical limitations and simultaneously determine patients' status. The dispersion coefficient is a strong AD marker that can separate AD EEG from MCI and HC.

### 4.2. Implementation of the Proposed Pattern Detection Method

In this research, the automatic classification of normal and abnormal EEG signals was built in a deep learning model. EEG signals are used in the EEG database. Documents are separated into two sections of the EEG database: training and testing samples. During the learning stage, the training data were used, and during the evaluation stage, assessment data were used for training the algorithms with 80% used as validation data, while the remaining with 20%.

These data distributions have been randomly chosen. For validation purposes, many datasets have been used since the model parameter is set in several steps. However, experimental results with a specific random seed value are obtained to ensure that the model is reproducible and uniform.  Figure 6 provides a thorough description of the data considered for this work. The block diagram of the process is described in Figure 8. Based on the process, firstly, TD-PSD is used for feature extraction of input EEG signals. The results of feature extraction are the produced seven features of values from 256 EEG samples.

Regarding this fact, the number of input variables for each person reduced from 256 to 7 features. It not only reduced the number of inputs but also increased the classification process speed. Signals with the time-dependent value are needed to be transformed into a meaningful value. Therefore, these values are extracted features. Altogether, it is 64 persons for each category of MCI, AD, and HC that each one has seven features. Therefore, the input matrix for each category has 7 × 64 elements.

In the next step, the output features are used for classification methods. For achieving this purpose, three powerful traditional methods of classification of EEG signal and diagnosis of AD and MCI patients from HC or healthy people are used. Used methods include KNN, SVM, and LDA. All the methods are chosen from powerful machine learning techniques. The results of classification for mentioned methods are as follows (Figure 9). Figure 9 shows the confusion matrix of utilized methods of classification. The labeling (1, 2, and 3) illustrates MCI, AD, and HC, respectively. Based on the confusion matrix. The green values show the number of persons diagnosed correctly from 64 people. Based on Figure 9(a), from 64 patients who suffered from MCI, 51 of them (79.7%) are diagnosed correctly.

Moreover, for people with AD, the sensitivity of the KNN is 71.9% (46 out of 64 patients). Moreover, 62.5% (40 persons) of healthy samples are detected correctly. Based on the results, the lower row of the matrix illustrates the sensitivity of the methods for the classification of each category. Moreover, red %ages indicated miss rates of each class. The right column of the matrix represents the precision of the KNN technique. Based on the results, 63.7% of the MCI-diagnosed patients are classified correctly. Other precision values are depicted in the right column. Finally, the accuracy of the methods is presented in the lower-right corner of the matrix. Based on the result, the accuracy of KNN, SVM, and LDA approaches is 71.4%, 41.1%, and 43.8%, respectively. In other words, the accuracy of the KNN is higher than that of the other methods. On the other hand, SVM and LDA methods represent results with very low accuracy. It can be noticed that the classification with two categories of patients and healthy people illustrates higher accuracy in comparison with three categories.

In this paper, a novel deep learning process for the classification of EEG signals is introduced based on a CNN. The architecture of the presented method is illustrated in Figure 10. Input layer includes the following:

- Seven features of 64 people for each category of MCI, AD, and HC
- Input matrix 4D [7 × 1 × 1 × 192]
- Output matrix 1D [1 × 192]

The labeling (1, 2, and 3) illustrates MCI, AD, and HC, respectively, output matrix. The process of the classification using the presented CNN architecture is shown in Figure 11. The maximum accuracy for the process reached almost 100%, and the loss value decreased to almost zero.

The confusion matrix of the presented method is indicated in Figure 12 without uncertainty value. The confident value of the accuracy for the CNN approach is 82.3%. In detail, 85% of the MCI patients are detected correctly; however, 89.1% of the AD and 75% of the normal sample are diagnosed correctly. For comparison of the resulted model of CNN with other KNN, SVM, and LDA techniques, the ROC plot is depicted in Figure 13. Regarding Figure 13, the value of FP rate versus TP rate is depicted based on output classification scores. Based on this graph, if the values would be higher for the TP rate and lower for the FP rate, it is better than the other graphs.

Moreover, the area under the curve (AUC) is one of the criteria for the classification method's performance analysis. Based on Figure 13, the presented CNN outperforms other methods, and the KNN method is in the following priority. The LDA and SVM reached low AUC values (see Table 2). To conclude, it can be seen that the presented CNN architecture is better and more accurate than other classification methods. Based on Table 2, the best method for diagnosing AD patients from EEG signals is the presented architecture's CNN approach.

## 5. Conclusion

In this article, the TD-PSD approach is used for EEG signal feature extraction from three groups of MCI, AD, and HC test samples. The final features used in three conventional classification methods are registered: KNN, SVM, and LDA, and the effects are recorded. Finally, the CNN architecture is provided for AD patient classification. The findings are indicated using performance measurement. Data were obtained with a signal duration of 300 seconds and a sampling frequency of 1024 and 256 samples per second. To minimize the EEG background artifacts, it obtains 180 seconds for each signal (i.e., from 60 to 240 seconds), and it is translated to 256 samples per second. The EEG ability of human samples belonging to three groups, including AD, MCI, and HC, has been summarized. First, the TD-PSD method is utilized to feature input EEG signals based on the procedure. The results of the extraction of features are the generation of seven value characteristics from 256 EEG samples. For classification methods, the output features are used in the next step. Methods used include KNN, SVM, and LDA. All the strategies are picked from effective methods in machine learning.

Based on the findings, 51 of the 64 patients with MCI (79.7%) were correctly diagnosed. In comparison, the KNN sensitivity for AD persons is 71.9% (46 out of 64 patients). In comparison, 62.5% (40 individuals) of sound samples are appropriately classified. Also, 63.7% of the MCI diagnosed patients are appropriately categorized based on the findings. In comparison, KNN, SVM, and LDA methods have a precision of 71.4%, 41.1%, and 43.8%, respectively. The precision of KNN, in other words, is greater than that of other processes. Then, a new EEG signal classification architecture is implemented that is focused on a CNN. For the CNN approach, the accurate meaning of accuracy is 82.3%. 85% of MCI cases are accurately detected in-depth, but 89.1% of the AD and 75% of the healthy population are correctly diagnosed. The presented CNN outperforms other approaches based on performance, and the KNN approach is the next target. The LDA and SVM were at low AUC values. For potential outcomes, it is recommended to modify feature extraction with another EEG signal justification for classification with a lower number of features and training using the design provided.

## Figures and Tables

**Figure 1:** The block diagram of the TD-PSD feature extraction method for EEG signals.

**Figure 2:** A conventional sublayer in CNN.

**Figure 3:** The place of electrodes of EGG signals.

**Figure 4:** Plots of sampling from EEG signals for three categories of MCI, AD, and HC.

**Figure 5:** Time-frequency analysis of EEG signals for MCI patients.

**Figure 6:** Time-frequency analysis of EEG signals for AD patients.

**Figure 7:** Time-frequency analysis of EEG signals for HC samples.

**Figure 8:** Conceptual diagram of the process used in this paper.

**Figure 9:** Confusion matrix of classification methods: (a) KNN, (b) SVM, and (c) LDA.

**Figure 10:** The architecture of the CNN layer for classification Alzheimer's disease.

**Figure 11:** Accuracy and loss values for classification process of the presented CNN.

**Figure 12:** Confusion matrix of the presented CNN method for classification of patients suffering from Alzheimer's.

**Figure 13:** The ROC curve for the presented methods.

**Table 1:** Summary of machine learning method for brain disease diagnosis with EEG signal.

Author	Year	Disease	Feature extraction	Classification	Results
Xin et al. [80]	2021	Epilepsy	Dimensionality reduction principal component analysis (PCA)	Convolution SVM	The method's accuracy, sensitivity, and specificity reach up to 99.56%, 99.72%, and 99.52%, respectively

Aliyu and Lim [81]	2021	Epilepsy	Discrete wavelet transforms (DWT)	LSTM network	Reduction of the number of LSTM trainable parameters needed to achieve extreme accuracy

Tuncer [82]	2021	Epileptic seizure	Nonlinear textural feature extraction (Hamsi hash)	*k*-nearest neighborhood	This model has an accuracy in the EEG dataset of 99.20% for five classes and has 100.0% accuracy in other conditions

Cicalese et al. [83]	2020	AD	Pearson correlation coefficient-based feature selection (PCCFS)	LDA	The EEG-fNIRS feature set combination was expected to obtain greater precision (79.31%) by combining its supplementary properties as compared with the EEG (65.52%) or fNIRS alone (58.62%). Moreover, AD development is associated with the right and left parietal lobe

Ferri et al. [84]	2020	AD	rsEEG + sMRI	Low-resolution brain electromagnetic tomography (LORETA)	Classification accuracy of 80%, 85%, and 89% using rsEEG, sMRI, and rsEEG + sMRI features, respectively, discriminates against them

Trambaiolli et al. [85]	2017	AD	Feature selection (FS)	SVM classifier	Since eliminating 88.76 ± 1.12% of the initial elements, the filtered subset evaluator technique obtained the highest efficiency gain, both on a per-patient basis (91.18% accuracy) and on a per-epoch basis (85.29 ± 21.62%)

Nobukawa et al. [86]	2020	AD	Functional connectivity	SVM	A novel interpretation of neural network functions in healthy brains and unhealthy disorders can be provided by applying a mixture of both machine learning approaches to neurophysiological evidence

Kulkarni and Bairagi [87]	2017	AD	Extracting salient features that are spectral-, wavelet-, and complexity-based	SVM	The increased performance in AD diagnosis

Vecchio et al. [88]	2020	AD	—	SVM	A low-cost and noninvasive process uses readily available tools that, when integrated, achieve high sensitivity/specificity and optimum individual classification accuracy (0.97 of AUC)

**Table 2:** Comparison of the diagnosis methods used in this paper.

	Sensitivity			Precision			AUC	Accuracy
	MCI	AD	HC	MCI	AD	HC		
KNN	79.7%	71.9%	62.5%	63.7%	75.4%	78.4%	0.902	71.4%
SVM	9.4%	32.8%	81.3%	31.6%	47.7%	40.3%	0.593	41.1%
LDA	28.1%	53.1%	50.0%	45.0%	43.0%	48.8%	0.594	43.8%
Presented CNN	82.8%	89.1%	75.5%	81.5%	79.2%	87.3%	0.988	82.3%

## Data Availability

Data is extracted from the following ref: An integrated approach based on EEG signals processing combined with supervised methods to classify Alzheimer's disease patients.

## References

[1] World Health Organization (2012). *Alzheimer's Disease International. Dementia: A Public Health Priority*.

[2] Duthey B. (2013). Background paper 6.11: Alzheimer disease and other dementias. *A Public Health Approach to Innovation*.

[3] Prince M., Wimo A., Guerchet M. (2015). The global impact of dementia: an analysis of prevalence, incidence, cost and trends. *Alzheimer's Disease International*.

[4] Lee E. E., Chang B., Huege S., Hirst J. (2018). Complex clinical intersection: palliative care in patients with dementia. *The American Journal of Geriatric Psychiatry*.

[5] Jack C. R., Albert M. S., Knopman D. S. (2011). Introduction to the recommendations from the National Institute on Aging-Alzheimer's Association workgroups on diagnostic guidelines for Alzheimer's disease. *Alzheimer's & Dementia*.

[6] McKhann G., Drachman D., Folstein M., Katzman R., Price D., Stadlan E. M. (1984). Clinical diagnosis of Alzheimer's disease: report of the NINCDS-ADRDA work group∗ under the auspices of department of health and human services task force on Alzheimer's disease. *Neurology*.

[7] Hort J., O’Brien J. T., Gainotti G. (2010). EFNS guidelines for the diagnosis and management of Alzheimer's disease. *European Journal of Neurology*.

[8] Folstein M. F., Folstein S. E., McHugh P. R. (1975). Mini-mental state: a practical method for grading the cognitive state of patients for the clinician. *Journal of Psychiatric Research*.

[9] Mitchell A. J. (2009). A meta-analysis of the accuracy of the mini-mental state examination in the detection of dementia and mild cognitive impairment. *Journal of Psychiatric Research*.

[10] Nasreddine Z. S., Phillips N. A., Bédirian V. (2005). The Montreal Cognitive Assessment, MoCA: a brief screening tool for mild cognitive impairment. *Journal of the American Geriatrics Society*.

[11] Mathuranath P. S., Nestor P. J., Berrios G. E., Rakowicz W., Hodges J. R. (2000). A brief cognitive test battery to differentiate Alzheimer's disease and frontotemporal dementia. *Neurology*.

[12] Amodio P., Wenin H., del Piccolo F. (2002). Variability of trail making test, symbol digit test and line trait test in normal people. A normative study taking into account age-dependent decline and sociobiological variables. *Aging Clinical and Experimental Research*.

[13] Shulman K. I. (2000). Clock-drawing: is it the ideal cognitive screening test?. *International Journal of Geriatric Psychiatry*.

[14] al-Qazzaz N. K., Ali S. H. B. M. D., Ahmad S. A., Chellappan K., Islam M. S., Escudero J. (2014). Role of EEG as biomarker in the early detection and classification of dementia. *The Scientific World Journal*.

[15] Montine T. J., Phelps C. H., Beach T. G. (2012). National Institute on Aging-Alzheimer's Association guidelines for the neuropathologic assessment of Alzheimer's disease: a practical approach. *Acta Neuropathologica*.

[16] Wu L., Wu L., Chen Y., Zhou J. (2014). A promising method to distinguish vascular dementia from Alzheimer's disease with standardized low-resolution brain electromagnetic tomography and quantitative EEG. *Clinical EEG and Neuroscience*.

[17] Dubois B., Feldman H. H., Jacova C. (2014). Advancing research diagnostic criteria for Alzheimer's disease: the IWG-2 criteria. *The Lancet Neurology*.

[18] Ferreira D., Perestelo-Pérez L., Westman E., Wahlund L. O., Sarría A., Serrano-Aguilar P. (2014). Meta-review of CSF core biomarkers in Alzheimer’s disease: the state-of-the-art after the new revised diagnostic criteria. *Frontiers in Aging Neuroscience*.

[19] Olsson B., Lautner R., Andreasson U. (2016). CSF and blood biomarkers for the diagnosis of Alzheimer's disease: a systematic review and meta-analysis. *The Lancet Neurology*.

[20] Seeck M., Koessler L., Bast T. (2017). The standardized EEG electrode array of the IFCN. *Clinical Neurophysiology*.

[21] Hu S., Lai Y., Valdes-Sosa P. A., Bringas-Vega M. L., Yao D. (2018). How do reference montage and electrodes setup affect the measured scalp EEG potentials?. *Journal of Neural Engineering*.

[22] Wang J., Barstein J., Ethridge L. E., Mosconi M. W., Takarae Y., Sweeney J. A. (2013). Resting-state EEG abnormalities in autism spectrum disorders. *Journal of Neurodevelopmental Disorders*.

[23] Faust O., Acharya U. R., Adeli H., Adeli A. (2015). Wavelet-based EEG processing for computer-aided seizure detection and epilepsy diagnosis. *Seizure*.

[24] Muniz C. F., Shenoy A. V., OʼConnor K. L. (2016). Clinical development and implementation of an institutional guideline for prospective EEG monitoring and reporting of delayed cerebral ischemia. *Journal of Clinical Neurophysiology*.

[25] Nishida K., Yoshimura M., Isotani T. (2011). Differences in quantitative EEG between frontotemporal dementia and Alzheimer's disease as revealed by LORETA. *Clinical Neurophysiology*.

[26] Jeong D.-H., Kim Y.-D., Song I.-U., Chung Y.-A., Jeong J. (2016). Wavelet energy and wavelet coherence as EEG biomarkers for the diagnosis of Parkinson's disease-related dementia and Alzheimer's disease. *Entropy*.

[27] Neto E., Allen E. A., Aurlien H., Nordby H., Eichele T. (2015). EEG spectral features discriminate between Alzheimer’s and vascular dementia. *Frontiers in Neurology*.

[28] Neto E., Biessmann F., Aurlien H., Nordby H., Eichele T. (2016). Regularized linear discriminant analysis of EEG features in dementia patients. *Frontiers in Aging Neuroscience*.

[29] Colloby S. J., Cromarty R. A., Peraza L. R. (2016). Multimodal EEG-MRI in the differential diagnosis of Alzheimer's disease and dementia with Lewy bodies. *Journal of Psychiatric Research*.

[30] Garn H., Coronel C., Waser M., Caravias G., Ransmayr G. (2017). Differential diagnosis between patients with probable Alzheimer's disease, Parkinson's disease dementia, or dementia with Lewy bodies and frontotemporal dementia, behavioral variant, using quantitative electroencephalographic features. *Journal of Neural Transmission*.

[31] Nunez P. L., Srinivasan R. (2006). *Electric Fields of the Brain: The Neurophysics of EEG*.

[32] Cohen M. (2014). *Analyzing Neural Time Series Data: Theory and Practice*.

[33] Sörnmo L., Laguna P. (2005). *Bioelectrical Signal Processing in Cardiac and Neurological Applications*.

[34] Dauwels J., Srinivasan K., Ramasubba Reddy M. (2011). Slowing and loss of complexity in Alzheimer's EEG: two sides of the same coin?. *International Journal of Alzheimer's Disease*.

[35] Alberdi A., Aztiria A., Basarab A. (2016). On the early diagnosis of Alzheimer's disease from multimodal signals: a survey. *Artificial Intelligence in Medicine*.

[36] Malek N., Baker M. R., Mann C., Greene J. (2017). Electroencephalographic markers in dementia. *Acta Neurologica Scandinavica*.

[37] Adeli H., Ghosh-Dastidar S., Dadmehr N. (2005). Alzheimer's disease: models of computation and analysis of EEGs. *Clinical and EEG Neuroscience*.

[38] Jelles B., van Birgelen J. H., Slaets J. P., Hekster R. E., Jonkman E. J., Stam C. J. (1999). Decrease of non-linear structure in the EEG of Alzheimer patients compared to healthy controls. *Clinical Neurophysiology*.

[39] Jeong J., Kim S. Y., Han S. H. (1998). Non-linear dynamical analysis of the EEG in Alzheimer's disease with optimal embedding dimension. *Electroencephalography and Clinical Neurophysiology*.

[40] Jeong J., Chae J. H., Kim S. Y., Han S. H. (2001). Non-linear dynamic analysis of the EEG in patients with Alzheimer's disease and vascular dementia. *Journal of Clinical Neurophysiology*.

[41] Takahashi T. (2013). Complexity of spontaneous brain activity in mental disorders. *Progress in Neuro-psychopharmacology & Biological Psychiatry*.

[42] Yagyu T., Wackermann J., Shigeta M. (1997). Global dimensional complexity of multi-channel EEG in mild Alzheimer's disease and age-matched cohorts. *Dementia and Geriatric Cognitive Disorders*.

[43] Houmani N., Vialatte F. B., Latchoumane C., Jeong J., Dreyfus G. Stationary epoch-based entropy estimation for early diagnosis of Alzheimer's disease.

[44] Houmani N., Vialatte F. B., Dreyfus G. (2015). Epoch-based entropy for early screening of Alzheimer's disease. *International Journal of Neural Systems*.

[45] Aba'solo D., Hornero R., Espino P., Alvarez D., Poza J. (2006). Entropy analysis of the EEG background activity in Alzheimer's disease patients. *Physiological Measurement*.

[46] De Bock T. J., Das S., Mohsin M. Early detection of Alzheimer's disease using non-linear analysis of EEG via Tsallis entropy.

[47] Aba'solo D., Hornero R., Espino P., Poza J., Sanchez C. I., de la Rosa R. (2005). Analysis of regularity in the EEG background activity of Alzheimer's disease patients with approximate entropy. *Clinical Neurophysiology*.

[48] Pincus S. M. (2006). Approximate entropy as a measure of irregularity for psychiatric serial metrics. *Bipolar Disorders*.

[49] Escudero J., Aba'solo D., Hornero R., Espino P., Lopez M. (2006). Analysis of electroencephalograms in Alzheimer's disease patients with multiscale entropy. *Physiological Measurement*.

[50] Aba'solo D., Hornero R., Gomez C. (2006). Analysis of EEG background activity in Alzheimer's disease patients with Lempel-Ziv complexity and central tendency measure. *Medical Engineering & Physics*.

[51] Chen W., Lam Y. Y., Shen C. P., Sung H. Y., Chiu M. J., Lai F. Ultra-fast epileptic seizure detection using EMD based on multi-channel electroencephalogram.

[52] Pei G., Wu J., Chen D. (2018). Effects of an integrated neurofeedback system with dry electrodes: EEG acquisition and cognition assessment. *Sensors*.

[53] Swapna G., Swapna G., Swapna G., Suri J. S., Suri J. S. (2013). Automated EEG analysis of epilepsy: a review. *Knowledge-Based Systems*.

[54] Yan T., Wang W., Liu T. (2017). Increased local connectivity of brain functional networks during facial processing in schizophrenia: evidence from EEG data. *Oncotarget*.

[55] Chen G., Xie W., Bui T. D., Krzyzak A. (2017). Automatic epileptic seizure detection in EEG using nonsubsampled wavelet–Fourier features. *Journal of Medical and Biological Engineering*.

[56] Hamad A., Houssein E. H., Hassanien A. E., Fahmy A. A. A hybrid EEG signals classification approach based on grey wolf optimizer enhanced SVMs for epileptic detection.

[57] Subasi A., Kevric J., Abdullah Canbaz M. (2017). Epileptic seizure detection using hybrid machine learning methods. *Neural Computing and Applications*.

[58] Wang B., Yan T., Ohno S., Kanazawa S., Wu J. (2016). Retinotopy and attention to the face and house images in the human visual cortex. *Experimental Brain Research*.

[59] Ahmedt-Aristizabal D., Fookes C., Nguyen K., Denman S., Sridharan S., Dionisio S. (2018). Deep facial analysis: a new phase I epilepsy evaluation using computer vision. *Epilepsy & Behavior*.

[60] Acharya U. R., Oh S. L., Hagiwara Y., Tan J. H., Adeli H. (2018). Deep convolutional neural network for the automated detection and diagnosis of seizure using EEG signals. *Computers in Biology and Medicine*.

[61] Hussein R., Palangi H., Ward R., Wang Z. J. *Epileptic Seizure Detection: A Deep Learning Approach*.

[62] Kulkarni N., Bairagi V. (2018). *EEG-Based Diagnosis of Alzheimer Disease: A Review and Novel Approach for Feature Extraction and Classification Techniques*.

[63] Parvez M. Z., Paul M. (2017). Seizure prediction using undulated global and local features. *IEEE Transactions on Biomedical Engineering*.

[64] Najafabadi M. M., Villanustre F., Khoshgoftaar T. M., Wald R., Muharemagic E., Seliya N. (2015). Deep learning applications and challenges in big data analytics. *Journal of Big Data*.

[65] Lecun Y., Bengio Y., Hinton G. (2015). Deep learning. *Nature*.

[66] Coşkun M., Yildirim Ö., Uçar A., Demir Y. (2017). An overview of popular deep learning methods. *European Journal of Technic*.

[67] Günther J., Pilarski P. M., Helfrich G., Shen H., Diepold K. (2014). First steps towards an intelligent laser welding architecture using deep neural networks and reinforcement learning. *Procedia Technology*.

[68] LeCun Y., Boser B., Denker J. S. (1989). Backpropagation applied to handwritten zip code recognition. *Neural Computation*.

[69] Uçar A., Demir Y., Güzeliş C. (2017). Object recognition and detection with deep learning for autonomous driving applications. *Simulation*.

[70] Beser F., Kizrak M. A., Bolat B., Yildirim T. Recognition of sign language using capsule networks.

[71] Mnih V., Kavukcuoglu K., Silver D. (2015). Human-level control through deep reinforcement learning. *Nature*.

[72] Yildirim O., Tan R. S., Acharya U. R. (2018). An efficient compression of ECG signals using deep convolutional autoencoders. *Cognitive Systems Research*.

[73] Yildirim Ö. (2018). A novel wavelet sequence based on deep bidirectional LSTM network model for ECG signal classification. *Computers in Biology and Medicine*.

[74] Yıldırım O., Pławiak P., Tan R. S., Acharya U. R. (2018). Arrhythmia detection using deep convolutional neural network with long duration ECG signals. *Computers in Biology and Medicine*.

[75] Oh S. L., Hagiwara Y., Raghavendra U. (2020). A deep learning approach for Parkinson's disease diagnosis from EEG signals. *Neural Computing and Applications*.

[76] Hong X., Lin R., Yang C. (2019). Predicting Alzheimer's disease using LSTM. *IEEE Access*.

[77] Aghili M., Tabarestani S., Adjouadi M. Predictive modeling of longitudinal data for Alzheimer's disease diagnosis using RNNs.

[78] Razavi F., Tarokh M. J., Alborzi M. (2019). An intelligent Alzheimer's disease diagnosis method using unsupervised feature learning. *Journal of Big Data*.

[79] Padilla P., López M., Górriz J. M., Ramírez J., Salas-González D., Álvarez I. (2012). NMF-SVM based CAD tool applied to functional brain images for the diagnosis of Alzheimer's disease. *IEEE Transactions on Medical Imaging*.

[80] Xin Q., Hu S., Liu S., Ma X., Lv H., Zhang Y. D. (2021). Epilepsy EEG classification based on convolution support vector machine. *Journal of Medical Imaging and Health Informatics*.

[81] Aliyu I., Lim C. G. (2021). Selection of optimal wavelet features for epileptic EEG signal classification with LSTM. *Neural Computing and Applications*.

[82] Tuncer T. (2021). A new stable non-linear textural feature extraction method-based EEG signal classification method using substitution Box of the Hamsi hash function: Hamsi pattern. *Applied Acoustics*.

[83] Cicalese P. A., Li R., Ahmadi M. B. (2020). An EEG-fNIRS hybridization technique in the four-class classification of Alzheimer's disease. *Journal of Neuroscience Methods*.

[84] Ferri R., Babiloni C., Karami V. (2021). Stacked autoencoders as new models for an accurate Alzheimer's disease classification support using resting-state EEG and MRI measurements. *Clinical Neurophysiology*.

[85] Trambaiolli L. R., Spolaôr N., Lorena A. C., Anghinah R., Sato J. R. (2017). Feature selection before EEG classification supports the diagnosis of Alzheimer's disease. *Clinical Neurophysiology*.

[86] Nobukawa S., Yamanishi T., Kasakawa S., Nishimura H., Kikuchi M., Takahashi T. (2020). Classification methods based on complexity and synchronization of electroencephalography signals in Alzheimer's disease. *Frontiers in Psychiatry*.

[87] Kulkarni N. N., Bairagi V. K. (2017). Extracting salient features for EEG-based diagnosis of Alzheimer's disease using support vector machine classifier. *IETE Journal of Research*.

[88] Vecchio F., Miraglia F., Alù F. (2020). Classification of Alzheimer's disease with respect to physiological aging with innovative EEG biomarkers in a machine learning implementation. *Journal of Alzheimer's Disease*.

[89] Hjorth B. (1970). EEG analysis based on time domain properties. *Electroencephalography and Clinical Neurophysiology*.

[90] Khushaba R. N., Takruri M., Miro J. V., Kodagoda S. (2014). Towards limb position invariant myoelectric pattern recognition using time-dependent spectral features. *Neural Networks*.

[91] Wellekens V., Tyagi C. On desensitizing the Mel-Cepstrum to spurious spectral components for robust speech recognition.

[92] Childers D. G., Skinner D. P., Kemerait R. C. (1977). The cepstrum: a guide to processing. *Proceedings of the IEEE*.

[93] He J., Zhang D., Sheng X., Li S., Zhu X. (2014). Invariant surface EMG feature against varying contraction level for myoelectric control based on muscle coordination. *IEEE Journal of Biomedical and Health Informatics*.

[94] Krizhevsky A., Sutskever I., Hinton G. E. (2012). Imagenet classification with deep convolutional neural networks. *Advances in Neural Information Processing System*.

[95] Hassantabar S., Ahmadi M., Sharifi A. (2020). Diagnosis and detection of infected tissue of COVID-19 patients based on lung x-ray image using convolutional neural network approaches. *Chaos, Solitons & Fractals*.

[96] Milletari F., Navab N., Ahmadi S. A. V-net: fully convolutional neural networks for volumetric medical image segmentation.

[97] Zhang R., Bai L., Zhang J., Tian L., Li R., Liu Z. Convolutional LSTM networks for vibration-based defect identification of the composite structure.

[98] Liu R., Wei S., Zhao Y., Yang Y. (2018). Indexing of the CNN features for the large scale image search. *Multimedia Tools and Applications*.

[99] Park S. H., Goo J. M., Jo C. H. (2004). Receiver operating characteristic (ROC) curve: practical review for radiologists. *Korean Journal of Radiology*.

[100] Jasper H. H. (1958). The ten-twenty electrode system of the international federation. *Electroencephalography and Clinical Neurophysiology*.

